# Comparison of the Accuracy of Two Conventional Phenotypic Methods and Two MALDI-TOF MS Systems with That of DNA Sequencing Analysis for Correctly Identifying Clinically Encountered Yeasts

**DOI:** 10.1371/journal.pone.0109376

**Published:** 2014-10-16

**Authors:** Qiao-Ting Chao, Tai-Fen Lee, Shih-Hua Teng, Li-Yun Peng, Ping-Hung Chen, Lee-Jene Teng, Po-Ren Hsueh

**Affiliations:** 1 Departments of Laboratory Medicine, National Taiwan University Hospital, National Taiwan University College of Medicine, Taipei, Taiwan; 2 Department and Graduate Institute of Clinical Laboratory Sciences and Medical Biotechnology, National Taiwan University, Taipei, Taiwan; 3 Department of Graduate Institute of Biomedical Sciences, Chang Gung University, Tao-Yuan, Taiwan; 4 Bruker Taiwan Co., Ltd., Taipei, Taiwan; 5 Departments of and Internal Medicine, National Taiwan University Hospital, National Taiwan University College of Medicine, Taipei, Taiwan; Leibniz Institute for Natural Products Research and Infection Biology- Hans Knoell Institute, Germany

## Abstract

We assessed the accuracy of species-level identification of two commercially available matrix-assisted laser desorption ionization-time of flight mass spectrometry (MALDI-TOF MS) systems (Bruker Biotyper and Vitek MS) and two conventional phenotypic methods (Phoenix 100 YBC and Vitek 2 Yeast ID) with that of rDNA gene sequencing analysis among 200 clinical isolates of commonly encountered yeasts. The correct identification rates of the 200 yeast isolates to species or complex (*Candida parapsilosis* complex, *C. guilliermondii* complex and *C. rugosa* complex) levels by the Bruker Biotyper, Vitek MS (using in vitro devices [IVD] database), Phoenix 100 YBC and Vitek 2 Yeast ID (Sabouraud's dextrose agar) systems were 92.5%, 79.5%, 89%, and 74%, respectively. An additional 72 isolates of *C. parapsilosis* complex and 18 from the above 200 isolates (30 in each of *C. parapsilosis*, *C. metapsilosis*, and *C. orthopsilosis*) were also evaluated separately. Bruker Biotyper system could accurately identify all *C. parapsilosis* complex to species level. Using Vitek 2 MS (IVD) system, all *C. parapsilosis* but none of *C. metapsilosis*, or *C. orthopsilosis* could be accurately identified. Among the 89 yeasts misidentified by the Vitek 2 MS (IVD) system, 39 (43.8%), including 27 *C. orthopsilosis* isolates, could be correctly identified Using the Vitek MS Plus SARAMIS database for research use only. This resulted in an increase in the rate of correct identification of all yeast isolates (87.5%) by Vitek 2 MS. The two species in *C. guilliermondii* complex (*C. guilliermondii* and *C. fermentati*) isolates were correctly identified by cluster analysis of spectra generated by the Bruker Biotyper system. Based on the results obtained in the current study, MALDI-TOF MS systems present a promising alternative for the routine identification of yeast species, including clinically commonly and rarely encountered yeast species and several species belonging to *C. parapsilosis* complex, *C. guilliermondii* complex, and *C. rugosa* complex.

## Introduction

Invasive candidiasis and candidemia remain leading causes of morbidity and mortality in immunocompromised hosts, particularly among patients with hematological malignancies in intensive care units [1]–[5]. Optimal and early therapy has been shown to significantly reduce the incidence of morbidity and mortality in patients with invasive yeast infections and has been shown to be associated with an overall reduction in cost of hospital care for these patients [5]. Although *Candida albicans* remains the predominant agent responsible for healthcare-associated infections, non-*albicans Candida* species, such as *C. glabrata*, *C. parapsilosis* complex, *C. tropicalis*, *C. guilliermondii* complex, *C. dubliniensis, C. lusitaniae*, and *C. krusei* have emerged as significant opportunistic pathogens [2]–[4]. Given the inherently variable antifungal susceptibility profiles of different *Candida* species and the emergence of infections due to previously rarely identified *Candida* species, correct identification to the species level is necessary for clinicians to make informed therapeutic decisions [2]–[5]. Recently developed molecular identification methods have shown that several members of *Candida* species (e.g. *C. parapsilosis* complex, *C. guilliermondii* complex, and *C. rugosa* complex) belong to the same complex [6]–[8].

The technologies for identification of yeasts have improved significantly over the past several decades, with methods ranging from simple manual biochemical assays to automated biochemical methods to complicated nucleic acid-based assays [9]–[11]. Using conventional laboratory methods (manual and automated), identification of yeast species responsible for infection usually take two days to several weeks [9]. Additionally, some of the methods are not very accurate at identifying less commonly encountered species [9]. Although these advancements in molecular techniques have greatly enhanced our ability to identify yeasts, many of the methods are associated with increased costs, longer turn-around time, and, in some instances, the need for considerable expertise [9]–[11]. Given these issues, matrix-assisted laser desorption ionization-time of flight mass spectrometry (MALDI-TOF MS)-based systems present a promising alternative for the routine identification of yeast species [12]–[14]. These systems provide correct species identification, take only a few minutes to perform, and are relatively inexpensive to conduct [8], [12]–[14]. However, few studies reported the performance of identification of species among *C. parapsilosis* complex, *C. guilliermondii* complex, and *C. rugosa* complex by phenotypic methods and MALDI-TOF MS assays.

In this study, we assessed the accuracy of species-level identification of two commercially available MALDI-TOF MS systems (Bruker Biotyper and Vitek MS) and two conventional phenotypic methods (Phoenix 100 YBC, Vitek 2 Yeast ID) for the identification of clinical yeast isolates. Accuracy was determined by comparing the results of those techniques with the results of rDNA gene sequencing analysis. Clustering analysis of the spectra of *C. parapsilosis* complex, *C. guilliermondii* complex, and *C. rugosa* complex by the Bruker Biotyper system were also performed.

## Methods

### Yeast Isolates

A total of 272 isolates of yeasts, including 90 randomly selected blood culture isolates of *C. parapsilosis* complex, were included in this study. These isolates included 91 challenge isolates provided by Becton-Dickinson Diagnostic Systems (Sparks, MD, USA) and 181 non-duplicate and randomly selected clinical isolates from patients who were treated at the National Taiwan University Hospital (NTUH) (Table 1). There were no differences in species distribution of yeasts between BD challenge isolates and NTUH isolates. All the *Candida* isolates collected from the NTUH were recovered from blood specimens from patients with candidemia. A total of 20 isolates of *Cryptococcus* species were recovered from blood (n = 10) and cerebrospinal fluid (n = 10). The other yeasts were isolated from various clinical specimens from patients treated at the NTUH. Among 90 isolates of *C. parapsilosis* complex, 18 isolates were randomly selected and included in the initial evaluation by four systems to reflect of common population distribution of different *Candida* species of the hospitals [1]–[4]. All the yeast isolates from the hospital (NTUH) and the 91 challenge strains from BD were subcultured twice from original stock solution to get the pure cultures (no mixed cultures) and were identified simultaneously by two commercial phenotypical methods, two MALDI-TOF MS methods, and molecular methods from the same culture plates these isolates grew. When any discordant results among isolates by these four phenotypical methods and molecular methods occurred, we repeated the identification methods to all the isolates (with discordant results) simultaneously.

**Table 1:** Identification results of 200 clinical isolates of yeasts by two commercial identification systems (Phoenix and Vitek 2 systems) and two MALDI-TOF MS systems (Bruker Biotyper and Vitek MS).

Species	No. of isolates tested (no. of BD challenge isolates)	No. (%) of isolates with identical identification results compared with those by gene sequencing analysis					
		Phoenix 100 YBC		Vitek 2 Yeast ID		MALDI-TOF MS	
		BAP	SDA	BAP	SDA	Bruker Biotyper	Vitek MS (CU database)
***Candida*** ** species**	**142**	**131 (92.2)**	**133 (93.7)**	**118 (83.1)**	**118 (83.1)**	**140 (98.6)**	**124 (87.3)**
*C. albicans*	19 (9)	19 (100)	19 (100)	18 (94.7)	19 (100)	19 (100)	19 (100)
*C. glabrata*	19 (10)	19 (100)	19 (100)	19 (100)	19 (100)	19 (100)	19 (100)
*C. parapsilosis* complex	18 (7)	18 (100)	18 (100)	18 (100)	18 (100)	18 (100)	6 (33.3)
*C. guilliermondii* complex	18 (7)	**17** (94.4)	16 (88.9)	**8** (44.4)	**5** (27.8)	18 (100)	**17** (94.4)
*C. tropicalis*	17 (7)	16 (94.1)	17 (100)	17 (100)	17 (100)	17 (100)	17 (100)
*C. krusei*	14 (8)	13 (92.9)	14 (100)	10 (71.4)	13 (92.9)	14 (100)	14 (100)
*C. dubliniensis*	6 (4)	6 (100)	5 (83.3)	6 (100)	5 (83.3)	6 (100)	6 (100)
*C. lusitaniae*	6 (1)	6 (100)	6 (100)	6 (100)	5 (83.3)	6 (100)	6 (100)
*C. rugosa* complex	4 (1)	3 (75)	4 (100)	3 (75)	3 (75)	4 (100)	3 (75)
*C. rugosa*	3 (0)	2 (66.7)	3 (100)	3 (100)	3 (100)	3 (100)	3 (100)
*C. pararugosa*	1 (0)	1 (100)	1 (100)	0 (0)	0 (0)	1 (100)	0 (0)
*C. kefyr*	3 (3)	3 (100)	3 (100)	2 (66.7)	2 (66.7)	3 (100)	3 (100)
*C. ciferrii*	2 (2)	2 (100)	2 (100)	2 (100)	2 (100)	2 (100)	2 (100)
*C. pelliculosa*	2 (2)	2 (100)	2 (100)	2 (100)	2 (100)	2 (100)	2 (100)
*C. nivariensis*	2 (1)	0 (0)	0 (0)	0 (0)	0 (0)	2 (100)	0 (0)
*C. utilis*	2 (1)	2 (100)	2 (100)	2 (100)	2 (100)	2 (100)	2 (100)
*C. catenulata*	1 (1)	1 (100)	1 (100)	1 (100)	1 (100)	1 (100)	1 (100)
*C. haemulonis*	1 (0)	1 (100)	1 (100)	1 (100)	1 (100)	1 (100)	1 (100)
*C. intermedia*	1 (0)	0 (0)	0 (0)	1 (100)	1 (100)	1 (100)	1 (100)
*C. pulcherrima*	1 (1)	1 (100)	0 (0)	0 (0)	0 (0)	1 (100)	1 (100)
*C. sphaerica*	1 (1)	0 (0)	1 (100)	0 (0)	1 (100)	1 (100)	1 (100)
C. *viswanathii*	1 (1)	1 (100)	1 (100)	0 (0)	0 (0)	0 (0)	0 (0)
*C. lipolytica*	1 (1)	1 (100)	1 (100)	1 (100)	1 (100)	1 (100)	1 (100)
*C. norvegensis*	1 (0)	0 (0)	1 (100)	1 (100)	1 (100)	1 (100)	1 (100)
C. *zeylanoides*	2 (2)	0 (0)	0 (0)	0 (0)	0 (0)	1 (50)	1 (50)
***Cryptococcus*** ** species**	**20**	**19 (95.0)**	**18 (90.0)**	**15 (75.0)**	**15 (75.0)**	**17 (85.0)**	**14 (70.0)**
*C. neoformans*	17 (7)	17 (100)	17 (100)	14 (82.4)	15 (88.2)	17 (100)	13 (76.5)
*C. albidus*	1 (1)	1 (100)	1 (100)	1 (100)	0 (0)	0 (0)	0 (0)
*C. humicolus*	1 (1)	1 (100)	0 (0)	0 (0)	0 (0)	0 (0)	1 (100)
*C. arboriformis*	1 (0)	0 (0)	0 (0)	0 (0)	0 (0)	0 (0)	0 (0)
*Rhodotorula mucilaginosa*	13 (2)	10 (76.9)	10 (76.9)	0 (0)	0 (0)	10 (76.9)	10 (76.9)
***Trichosporon*** ** species**	**8**	**5 (62.6)**	**7 (87.5)**	**7 (87.5)**	**6 (75)**	**6 (75)**	**5 (62.5)**
*T. asahii*	6 (0)	4 (66.7)	6 (100)	6 (100)	5 (83.3)	5 (83.3)	5 (83.3)
*T. mucoides*	1 (1)	1 (100)	1 (100)	1 (100)	1 (100)	1 (100)	0 (0)
*T. insectorum*	1 (0)	0 (0)	0 (0)	0 (0)	0 (0)	0 (0)	0 (0)
***Pichia*** ** species**	**2 (0)**	**0 (0)**	**2 (0)**	**1 (50.0)**	**1 (50.0)**	**1 (50.0)**	**1 (50.0)**
*P. norvegensis*	1 (0)	0 (0)	0 (0)	1 (100)	1 (100)	1 (100)	1 (100)
*P. fabianii*	1 (0)	0 (0)	0 (0)	0 (0)	0 (0)	0 (0)	0 (0)
*Saccharomyces cervevisiae*	5 (4)	5 (100)	5 (100)	5 (100)	5 (100)	5 (100)	5 (100)
*Prototheca wickerhamii*	2 (2)	2 (100)	2 (100)	2 (100)	2 (100)	2 (100)	0 (0)
*Lodderomyces elongisporus*	2 (0)	0 (0)	0 (0)	0 (0)	0 (0)	2 (100)	0 (0)
*Sporobolomyce salmonicolor*	2 (1)	1 (50)	1 (50)	0 (0)	0 (0)	2 (100)	0 (0)
*Thermus scotoductus*	1 (0)	0 (0)	0 (0)	0 (0)	0 (0)	0 (0)	0 (0)
*Geotrichum klebahnii*	1 (1)	0 (0)	0 (0)	1 (100)	1 (100)	0 (0)	0 (0)
*Hortaea werneckii*	1 (1)	0 (0)	0 (0)	0 (0)	0 (0)	0 (0)	0 (0)
*Rhodosporidium toruloides*	1 (0)	0 (0)	0 (0)	0 (0)	0 (0)	0 (0)	0 (0)
**Overall**	**200 (91)**	**173 (86.5)**	**178 (89)**	**149 (74.5)**	**148 (74.0)**	**185 (92.5)**	**159 (79.5)**

**Note.** BAP: trypticase soy agar with 5% sheep blood agar plates. SDA: Sabouraud dextrose agar. CU: clinical use.

The study was reviewed and approved by the institutional Review Board of National Taiwan University Hospital (number 201211073RSC) with waiver of requirement for obtaining informed consent. Patient-related data associated with the yeast isolates, i.e., age and sex of the patients, are not presented for ethical considerations. No verbal or written informed consent was obtained from the patients in this study.

### Phenotypic Characteristics of Isolates

Species identification was performed using the Vitek 2 yeast identification card (Vitek 2 Yeast ID; bioMérieux, Marcy l'Etoile, France) and Phoenix 100 Yeast ID panel (Becton-Dickinson Microbiology Systems, Sparks, MD, USA), according to the manufacturer's instructions [15]. Prior to testing, the isolates were subcultured onto Sabouraud dextrose agar (SDA, bioMérieux) and trypticase soy agar on 5% sheep blood agar plates (BAP, BD Microbiology System) and were incubated at 35°C in an aerobic atmosphere for 24–48 h. Extended incubation to 72 h was needed to ascertain adequate growth. *C. albicans* ATCC 14053 (Vitek 2 YST), *C. albicans* ATCC 24433, and *C. parapsilosis* ATCC 22019 (Phoenix Yeast ID panel) were used as control strains.

### Performance of Bruker Biotyper

For analysis of the 272 yeast isolates by the MALDI-TOF Biotyper (Bruker Biotyper) system, samples were prepared as previously described [16]. A single colony from a BAP (BD Microbiology System) was subjected to an ethanol-formic acid extraction procedure for microorganism profiling. Briefly, two to three yeast colonies were transferred using a 5-µl inoculating loop into 300 µl of distilled water and 900 µl of ethanol. The suspension was pelleted after centrifugation at 12,000 rpm for 2 min, dried, and then reconstituted in 50 µl of 70% formic acid. After incubation for 30 seconds, 50 µl of acetonitrile (Sigma-Aldrich) was added. The suspension was then centrifuged at 12,000 rpm for 2 min. A volume of 1.0 µl of the supernatant was applied to a 96-spot polished steel target (Bruker Daltonik GmbH, Bremen, Germany) plate and dried. A saturated solution of 1.0 ml of MALDI matrix (HCCA; Bruker Daltonik) was applied to each sample and dried. Measurements were performed with Bruker Microflex LT MALDI-TOF MS (Bruker Daltonik GmbH) using FlexControl software with Compass Flex Series version 1.3 software and a 60 Hz nitrogen laser (337 nm wavelength). Spectra were collected in the linear positive mode in a mass range covering 1,960 to 20,132 m/z. Spectra ranging from the mass-to-charge ratio (m/z) 2,000 to 20,000 were analyzed using MALDI Biotyper automation control and the Bruker Biotyper 3.1 software and library (version 3.1.66, with 4,613 entries; Bruker Daltonics). Identification scores of ≥2.000 indicated species-level identification, scores of 1.700 to 1.999 indicated genus-level identification, and scores of <1.700 indicated no identification.

### Cluster Analysis by Bruker Biotyper for *C. parapsilosis* Complex, *C. guilliermondii* Complex, and *C. rugosa* Complex Isolates

Clustering analysis of the isolates was performed using ClinProtools 3.0 (Bruker Daltonics GmbH, Bremen, Germany). *C. parapsilosis* complex, *C. guilliermondii* complex, and *C. rugosa* complex were analyzed for specific signals by clustering analysis [17]. In this study, there were 90 isolates of *C. parapsilosis* complex, including 30 isolates of *C. parapsilosis*, 30 isolates of *C. metapsilosis*, and 30 isolates of *C. orthopsilosis*. There were 18 isolates of *C. guilliermondii* complex, including 13 isolates of *C. guilliermondii* and five isolates of *C. fermentati*. In addition, four isolates of *C. rugosa* complex, including three *C. rugosa* and one *C. pararugosa* isolates.

### Performance of the Vitek MS System

Samples of the 272 yeast isolates were prepared for analysis by the Vitek MS system as reported previously with slight modifications [16]. Briefly, a 1-µl loop (Sarstedt, Newton, NC) was used to apply a portion of a single colony to a disposable target slide (bioMérieux) composed of a polypropylene carrier. Formic acid (0.5 µl, 25% [vol/vol]; bioMérieux) was then applied directly to the isolate immediately after application on the target plate. The formic acid overlay was allowed to dry at room temperature. Then 1 µl of CHCA matrix solution (3.1% [wt/vol] α-cyano-4-hydroxycinnamic acid; bioMérieux) was applied and allowed to dry at room temperature prior to mass spectrometric analysis. The isolate information was transferred to the Vitek MS acquisition station using Myla v3.2 middleware. The samples were analyzed with the Vitek MS in linear positive-ion mode across the mass-to-charge ratio range of 2,000 to 20,000 Da. The resulting quantitative value (confidence value) was then calculated and expresses the similarity between the unknown yeast and every yeast or yeast group in the two database systems (MS-ID version 2.0 knowledge base clinical use or in vitro devices [IVD] and Vitek MS Plus SARAMIS Knowledge Base Version 4.10 for research use only (RUO) (if the isolates were identified or reported as no identification in the database for CU). A single identification is displayed (green), with a confidence value (% probability) from 60.0 to 99.9 (good confidence level), when one significant yeast or yeast group is retained. “Low-discrimination” identifications are displayed (red) when two to four significant yeasts or yeast groups are retained. When more than four yeasts or yeast groups are found, or when no match is found, the yeast is considered un-identified (orange). Freshly prepared *Escherichia coli* ATCC 8739, *Enterococcus faecalis* ATCC 19433, and *C. glabrata* ATCC MYA 2950 were used as control strains.

### Molecular Identification

For sequence analysis of the isolates, two fungus-specific universal primers were used to amplify the region spanning the internal transcribed spacer region of the 5.8S rRNA gene (5′-TCC GTAGGTGAACCTGCGG-3′) and the internal transcribed spacer region of the 18S and 28S rRNA genes (5′-TCCTCCGCTTATTGATATGC-3′) [11]. For species identification of *Trichosporon* species, sequences of the ribosomal DNA IGS1 region, which is located between the 26S and 5S rRNA genes, were also analyzed [18]. The IGS1 region (which ranges in length from 195 to 719 bp) was amplified using the primers 26SF (5′-ATCCTTTGCAGACGACTTGA-3′) and 5SR (5′-AGCTTGACTTCGCAGATCGG-3′) [18]. The determined sequence was then compared with sequences available in GenBank by means of the BLAST program (http://blast.ncbi.nlm.nih.gov/Blast.cgi). Results were considered acceptable if homology with other entries in the databases used for comparison was >99.5%. *C. guilliermondii* complex isolates were further subjected to PCR with the primers RIBO-F (5′-ACAGTTGGTCGAGGTGGTC-3′) and RIBO-R (5′-CCTGGGTTCCCAAGTAGTCA-3′) for the riboflavin synthetase gene [7]. The amplified products were cleaved by restriction enzyme *Hga*I or *Hinc*II to differentiate between *C. guilliermondii* and *C. fermentati. C. guilliermondii* BCRC22093 (ATCC 46036), *C. fermentati* BCRC23164, and (CBS9966) were used as control strains.

### Statistical Analysis

The chi-square test was used to evaluate the performance of two conventional phenotypic methods (Phoenix 100 YBC, Vitek 2 Yeast ID) and two commercially available MALDI-TOF MS systems (Bruker Biotyper and Vitek MS) for the identification of all isolates of *Candida* species, *Cryptococcus* species, and all yeast isolates. *P* values <0.05 are considered statistically significant.

## Results

### Yeast Isolates

Of the 272 isolates of yeast species confirmed by DNA sequencing analysis, 214 were *Candida* species, 20 were *Cryptococcus* species, 13 were *Rhodotorula mucilaginosa*, 8 were *Trichosporon* species, 5 were *Saccharomyces cervevisiae*, 2 were *Pichia* species and the remaining 10 isolates were unusual species. The sequencing results had >99.5% homology with other entries in the databases. Among the 90 isolates of C. *parapsilosis* complex, all were subjected to cluster analysis by the Bruker Biotyper system and 18 randomly selected isolates were used for assessment of the accuracy of two commercially available MALDI-TOF MS systems and two conventional phenotypic methods.

### Results of DNA Sequencing Compared with those of Vitek 2 Yeast ID and Phoenix 100 YBC

Table 1 shows the number and proportions of the 200 yeast isolates that were correctly identified by the Phoenix YBC system and the Vitek 2 Yeast ID system on SDA and BAP. Overall, the performance of both systems on SDA and BAP was similar for *Candida* species (*P* = 0.640 for Phoenix YBC system and *P* = 1.000 for Vitek 2 Yeast ID system) and all yeast isolates (*P* = 0.445 for Phoenix YBC system and *P* = 0.909 for Vitek 2 Yeast ID system). The correct identification rates of the 200 isolates to the species or complex (*C. parapsilosis* complex, *C. guilliermondii* complex, and *C. rugosa* complex) levels on SDA by the Phoenix 100 was better than that by Vitek 2 Yeast ID systems (89.0% vs. 74.0%; *P*<0.001), respectively. For 142 isolates of *Candida* species, the Phoenix 100 YBC (SDA) and Vitek 2 Yeast ID (SDA) systems correctly identified 93.7% (n = 133) and 83.1% (n = 118) (*P* = 0.005), respectively, of the isolates to the species or complex levels. Neither system was able to correctly identify species among isolates of *C. parapsilosis* complex and *C. guilliermondii* complex. Using the Vitek 2 Yeast ID system, one *C. albicans* isolate was identified as C. *albicans*/C. *famata* on BAP. In addition, four isolates of *C. krusei* on BAP and one on SDA were reported as *C. krusei/C. lambica/C. inconspicua* (Table 2). The majority of misidentified species among *C. guilliermondii* complex isolates were *C. famata* or *C. famata/C. guilliermondii*. (Table 2). *Kodamaea ohmeri* was identified both on the BAP and SDA by the Vitek 2 system and *C. guilliermondii* var. *membranaefaciens* was identified on BAP by Phoenix 100 YBC system. Because *K. ohmeri* is an ascosporogenous yeast and a teleomorph of *C. guilliermondii* var. *membranaefaciens*, both identifications were considered correct as *C. guilliermondii* complex.

**Table 2:** Identification results of clinical isolates of yeasts by two commercial identification systems (Phoenix and Vitek 2 systems) and two MALDI-TOF MS systems (Bruker Biotyper and Vitek MS).

Species	No. of isolates tested	Species with misidentified results by indicated method compared with those by gene sequencing analysis (no. of isolates)					
		Phoenix 100 YBC		Vitek 2 Yeast ID		MALDI-TOF MS	
		BAP	SDA	BAP	SDA	Biotyper	Vitek MS (CU database)
***Candida*** ** species**							
*C. albicans*	19	-	-	C.*albicans*/C. *famata* (1)	-	-	-
*C. guilliermondii* complex	18	Unidentified (1)	C. *albicans* (1), C. *melibiosica* (1)	*C. famata* (4)*C. sphaerica* (1), C. *famata*/*C. guilliermondii* (5)	*C. famata* (3), C. *famata*/*C. guilliermondii* (10)	-	*C. famata* (1)
*C. tropicalis*	17	C. *viswanathii* (1)	-	-	-	-	-
*C. krusei*	14	C. *apicola* (1)	-	*C. krusei/C. lambica/C. inconspicua* (4)	*C. krusei/C. lambica/C. inconspicua* (1)	-	-
*C. dubliniensis*	6	-	*C. albicans* (1)	-	*C. krusei*/*C. dubliniensis* (1)	-	-
*C. lusitaniae*	6	-	-	-	C. *famata*/C. *lusitaniae*/C. *tropicalis* (1)	-	-
*C. rugosa*	1	No ID (1)	-	*-*	*-*	-	-
*C. pararugosa*	1	-	-	*Candida sphaerica* (1)	*C. rugosa/Geotrichum klebahnii* (1)	-	No ID (1)
*C. kefyr*	3	-	-	*C. sphaerica* (1)	*C. sphaerica* (1),	-	-
*C. nivariensis*	2	*C. glabrata* (1), Unidentified (1)	*C. glabrata* (1), *Zygosaccharomyces bailli* (1)	*C. glabrata* (2)	*C. glabrata* (1), No ID (1)	-	*C. glabrata* (1), *Pichia angusta* (1)
*C. intermedia*	1	*C. tropicalis* (1)	*C. melibiosica* (1)	-	-	-	-
*C. pulcherrima*	1	-	No ID (1)	Unidentified (1)	No ID (1)	-	-
*C. sphaerica*	1	Unidentified (1)	-	*C. pulcherrima* (1)	-	-	-
C. *viswanathii*	1	-	-	*C. tropicalis* (1)	No ID (1)	*C. tropicalis* (1)	*C. tropicalis* (1)
*C. norvegensis*	1	*P. farinose* (1)	-	-	-	-	-
C. *zeylanoides*	2	*S. cerevisiae* (1), *Trichosporon asahii* (1)	*S. cerevisiae* (1), *T. asahii* (1)	*S. cerevisiae* (1), *T. asahii* (1)	*S. cerevisiae* (1), *T. asahii* (1)	*C. robusta* (1)	*T. asahii* (1)
***Cryptococcus species***	**20**						
*C. neoformans*	17	-	-	*C. laurentii/C. neoformans* (2), C. *laurentii* (1)	C. *laurentii* (2)	-	No ID (4)
*C. albidus*	1	-	-	-	C. *laurentii/Rhodotorula* (1)	No ID (1)	No ID (1)
*C. humicolus*	1	-	No ID (1)	*C. lipolytica* (1)	*C. glabrata* (1)	*Filifactor villosum* (1)	*-*
*C. arboriformis*	1	No ID (1)	*T. inkin* (1)	S. *ciferrii* (1)	*Stephanoascus ciferrii* (1)	No ID (1)	*Prototheca zopfii* (1)
*Rhodotorula mucilaginosa*	**13**	*P. wickerhamii* (2), *S. cerevisiae* (1)	*P. wickerhamii* (2), *S. cerevisiae* (1)	*C. laurentii/R. mucilaginosa*/*R. glutinis* (10), *P. wickerhamii* (2), *S. cerevisiae* (1)	*C. laurentii/R. mucilaginosa/R. glutinis* (10), *P. wickerhamii* (2), *S. cerevisiae* (1)	*P. wickerhamii* (2), *C. tropicalis* (1)	*C. albidus* (1), No ID (2)
***Trichosporon*** ** species**	**8**						
*T. asahii*	6	*C. neoformans* (1)	-	-	*C. laurentii* (1)	No ID (1)	*Trichosporon asteroids* (1)
*T. mucoides*	1	-	-	-	-	-	*Geotrichum klebahnii* (1)
*T. insectorum*	1	No ID (1)	No ID (1)	*T. asahii* (1)	*T. asahii* (1)	*C. albicans* (1)	*T. asteroides* (1)
***Pichia*** ** species**	**8**						
*P. norvegensis*	1	*P. farinose* (1)	*C. firmetaria* (1)	-	-	-	-
*P. fabianii*	1	*Candida utilis* (1)	*P. burtonii* (1)	*C. utilis* (1)	*C. utilis* (1)	No ID (1)	No ID (1)
*Saccharomyces cervevisiae*	**5**						
*Prototheca wickerhamii*	2	-	-	-	-	-	No ID (2)
*Lodderomyces elongisporus*	2	*P. zopfii* (1), Unidentified (1)	*C. albicans* (2)	*C. parapsilosis* (2)	*C. parapsilosis* (2)	-	*C. pelliculosa* (2)
*Sporobolomyces salmonicolor*	2	*S. cerevisiae* (1)	S. cerevisiae (1)	*S. cerevisiae* (1), *C. laurentii/R. mucilaginosa/R. glutinis* (1)	*S. cerevisiae* (1), *C. laurentii/R.mucilaginosa/R. glutinis* (1)	-	*S. cerevisiae* (1), No ID (1)
*Thermus scotoductus*	1	*C. neoformans* (1)	*C. albidus* (1)	*C. albidus* (1)	*C. albidus* (1)	*C. neoformans* (1)	No ID (1)
*Geotrichum klebahnii*	1	*Geotrichum* species (1)	*Geotrichum* species (1)	-	-	*Geotrichum. candidum* (1)	*G. candidum* (1)
*Hortaea werneckii*	1	No ID (1)	No ID (1)	*C. lipolytica/C. famata/C. sake* (1)	*C. lipolytica/C. famata/C. sake* (1)	No ID (1)	No ID (1)
*Rhodosporidium toruloides*	1	*R. mucilaginosa var mucilaginosa* (1)	*R. mucilaginosa var mucilaginosa* (1)	*C. laurentii/R. mucilaginosa/R. glutinis* (1)	*C. laurentii/R. mucilaginosa/R. glutinis* (1)	*R. glutinis* (1)	*R. glutinis* (1)

**Note.** BAP: trypticase soy agar with 5% sheep blood agar plates. IVD: in vitro devices. No ID, no identification. SDA: Sabouraud dextrose agar.

For *Cryptococcus* isolates, 90.0% (n = 18) were correctly identified to the species level by the Phoenix 100 YBC system and 75.0% (n = 15) were correctly identified to the species level by the Vitek 2 Yeast ID (SDA) system (*P* = 0.210). When using the Phoenix system for identification of *Trichosporon* species, we found that SDA resulted in a better identification rate than BAP (87.5% vs. 62.6%). Of the 13 isolates of *Rhodotorula mucilaginosa*, 76.9% could be accurately identified to the species level by the Phoenix 100 YBC system; however, none of the isolates were correctly identified using the Vitek 2 Yeast ID system.

### Results of DNA Sequencing Compared with those of the Bruker Biotyper and Vitek MS Systems

Overall, the correct identification rates for all 200 yeast isolates were 92.5% for the Bruker Biotyper system and 79.5% for the Vitek MS (IVD database) system (*P*<0.001). For *Candida* species isolates, 98.6% (10.0% [n = 14] with score values of 1.800–1.994 and 90.0% [n = 126] with score values of 2.019–2.428) were correctly identified by Bruker Biotyper system and 87.3% (all with confidence values of 99.9%) by Vitek MS (IVD database) system (*P*<0.001) (Table 1). The low rate of correct identification of *C. parapsilosis* complex isolates to the species level by the Vitek MS system (IVD database) was due to the fact that 12 of the 18 *C. parapsilosis* complex isolates were *C. metapsilosis* (n = 6) and *C. orthopsilosis* (n = 6), which are not listed in the CU database. Among 90 isolates of *C. parapsilosis* complex, the Bruker Biotyper system was able to correctly identify all three species of *C. parapsilosis* (score value range, 1.996–2.241), *C. metapsilosis* (score value range, 1.731–2.271) and *C. orthopsilosis* (score value range, 1.701–2.086).

Vitek MS (CU database) failed to identify four isolates of *C. neoformans* and both systems failed to identify two other *Cryptococcus* species. For isolates of *Trichosporon*, the Vitek MS (IVD database) system also failed to accurately identify all of the isolates to the species level, including *T. asahii*. Both systems could adequately identify all *S. cervevisiae* isolates. The Bruker Biotyper but not the Vitek MS (IVD database) could correctly identify all isolates of *P. wickerhamii*, *Lodderomyces elongisporus*, and *Sporobolomyce salmonicolor* (Table 1).

Using the Vitek MS plus SARAMIS system (RUO database) to 89 initially misidentified yeast isolates, 39 isolates, including 27 of *C. orthopsilosis*, were correctly identified (Table 3). All the six *C. orthopsilosis* isolates in the 200 initially evaluated isolates were correctly identified by Vitek MS plus SARAMIS system RUO databases. This resulted in an increase in the rate of correct identification of all *Candida* species (94.3%, [134/142]) and all yeast isolates (87.5% [175/200]) tested by Vitek MS plus SARAMIS system RUO databases. There was no significant difference in the correct identification of all *Candida* species (*P* = 0.053) and all yeast isolates (*P* = 0.096) between Bruker Biotyper system and Vitek MS plus SARAMIS system RUO databases.

**Table 3:** Identification results using two Vitek MS databases, clinical use (CU) and Vitek MS Plus SARAMIS for research use only (RUO) for 89 yeast isolates initially misidentified or with no identification (No ID).

Species (identified by gene sequencing analysis)	No. of isolates	Vitek MS by IVD database (% probability)	Vitek MS Plus SARAMIS for RUO (% probability)
*C. metapsilosis*	27	No ID	No ID
	3	No ID	*C. parapsilosis* (44.6–55.3)
*C. orthopsilosis*	27	No ID	***C. orthopsilosis*** ** (75–96.2, n = 24) (54.6–58.6, n = 3)**
	2	*C. parapsilosis* (99.9)	*C. parapsilosis* (93.2–96.2)
	1	No ID	No ID
*C. guilliermondii* complex	1	*C. famata* (77)	***C. guilliermondii*** ** (99.9)**
*C. pararugosa*	1	No ID	*C. albicans* (99.9)
*C. nivariensis*	1	*C. glabrata* (87.6)	*C. glabrata* (87.6)
	1	*Pichia angusta* (99.9)	***C. nivariensis*** ** (99.9)**
C. *viswanathii*	1	*C. tropicalis* (99.9)	**C. ** ***viswanathii*** ** (54.8)**
C. *zeylanoides*	1	*Trichosporon asahii* (99.9)	**C. ** ***zeylanoides*** ** (96.6)**
*C. neoformans*	3	No ID	No ID
	1	No ID	***C. neoformans*** ** (99.9)**
*C. albidus*	1	No ID	No ID
*C. arboriformis*	1	*Prototheca zopfii* (85.5)	No ID
*Rhodotorula mucilaginosa*	1	*C. albidus* (97.1)	No ID
	2	No ID	No ID
*T. asahii*	1	*Trichosporon asteroids* (99.9)	No ID
*T. mucoides*	1	*Geotrichum klebahnii* (99.8)	No ID
*T. insectorum*	1	*Trichosporon asteroides* (99.9)	No ID
*Pichia fabianii*	1	No ID	***Pichia fabianii*** ** (99.9)**
*Prototheca wickerhamii*	1	No ID	No ID
	1	No ID	***Prototheca wickerhamii*** ** (99.9)**
*Lodderomyces elongisporus*	2	*C. pelliculosa* (84.4, 99.9)	***Lodderomyces elongisporus*** ** (99.9)**
*Sporobolomyce salmonicolor*	1	No ID	***Sporobolomyce salmonicolor*** ** (95.3)**
	1	*S. cerevisiae* (99.9)	***Sporobolomyce salmonicolor*** ** (99.9)**
*Thermus scotoductus*	1	No ID	No ID
*Geotrichum klebahnii*	1	*G. candidum* (99.9)	*G. klebahnii* (60.2)
*Hortaea werneckii*	1	No ID	No ID
*Rhodosporidium toruloides*	1	*R. glutinis* (99.9)	*R. glutinis* (75.2)

**Note.** Species typed in bold face indicate correct identification using Vitek MS Plus SARAMIS database for RUO for yeast isolates which were initially misidentified or reported no ID.

### Clustering Analysis of the Spectra of *C. parapsilosis* Complex, *C. guilliermondii* Complex, and *C. rugosa* Complex by the Bruker Biotyper System

The 90 isolates of *C. parapsilosis* complex were subjected to cluster analysis (Figures 1A and 1B). Ten peaks in the spectra of these isolates, i.e., 3380.19 *m/z*, 4,993.07 *m/z*, 5383.92 *m/z*, 5411.78 *m/z*, 5582.74 *m/z*, 5668.24 *m/z*, 7014.07 *m/z*, 7070.65 *m/z*, 7212.67 *m/z*, and 7326.88 *m/z* which were generated by ClinProTools with the genetic algorithm, were used to define clusters 1, 2, and 3 (Figures 1A and 1B). Three signals, namely 4,993.07 *m/z*, 5411.78 *m/z*, and 7070.65 *m/z*, were observed only in the cluster 1 spectrum (all were *C. parapsilosis*), three signals, namely 3380.19 *m/z*, 5383.92 *m/z*, and 7014.07 *m/z*, were observed only in the spectrum for cluster 2 (all were *C. orthopsilosis*), and four signals, namely 5582.74 *m/z*, 5668.24 *m/z*, 7212.67 *m/z*, and 7326,88 *m/z*, were observed only in the cluster 3 spectrum (all were *C. metapsilosis*).

**Figure 1:** Cluster analysis of MALDI-TOF Bruker Biotyper results for the 90 isolates of *C. parapsilosis* complex. **A.** Three clusters of *C. parapsilosis* complex spectra, i.e., cluster 1 (*C. parapsilosis*), cluster 2 (*C. orthopsilosis*), and cluster 3 (*C. metapsilosis*). **B.** The 10 peaks used to define cluster 1 (*C. parapsilosis*), cluster 2 (*C. orthopsilosis*), and cluster 3 (*C. metapsilosis*), which were generated by ClinProTools with the genetic algorithm, are 3380.19 *m/z*, 4,993.07 *m/z*, 5383.92 *m/z*, 5411.78 *m/z*, 5582.74 *m/z*, 5668.24 *m/z*, 7014.07 *m/z*, 7070.65 *m/z*, 7212.67 *m/z*, and 7326,88 *m/z*. Three signals 4,993.07 *m/z*, 5411.78 *m/z*, and 7070.65 *m/z* were observed only in the spectrum for cluster 1 (all were *C. parapsilosis*) spectra, three signals 3380.19 *m/z*, 5383.92 *m/z*, and 7014.07 *m/z* were observed only in the spectrum for cluster 2 (all were *C. orthopsilosis*) spectra, and four signals 5582.74 *m/z*, 5668.24 *m/z*, 7212.67 *m/z*, and 7326.88 *m/z* were observed only in the spectrum for cluster 3 (all were *C. metapsilosis*) spectra. The absolute intensities of the ions are shown on the *y* axis, and the masses (*m/z*) of the ions are shown on the *x* axis. The *m/z* values represent the mass-to-charge ratio. (C) Distribution of identification score values among three species of *C. parapsilosis* complex by MALDI-TOF Bruker Biotyper system.

As for the 18 isolates of *C. guilliermondii* complex (13 *C. guilliermondii* and five of *C. fermentati* isolates), five signals, i.e., 3181.57 *m/z*, 3359.10 *m/z*, 5218.25 *m/z*, 6717.05 *m/z*, and 6732.14 *m/z* were used to define clusters I and II (Figures 2A and 2B). Three signals, namely 3181.57 *m/z*, 5218.25 *m/z*, and 6732.14 *m/z*, were observed only in the spectrum for cluster I (all were *C. guilliermondii*) and two signals, 3359.10 *m/z* and 6717.05 *m/z*, were observed only in the spectrum for cluster II (all were *fermentati*) (Figures 2A and 2B).

**Figure 2:** Cluster analysis of MALDI-TOF Bruker Biotyper results for the 18 isolates of *C. guilliermondii* complex. **A.** Two clusters of *C. guilliermondii* complex spectra, i.e., cluster I (*C. fermentati*) and cluster II (*C. guilliermondii*). **B.** The five peaks used to define cluster I (*C. fermentati*) and cluster II (*C. guilliermondii*), which were generated by ClinProTools with the genetic algorithm, are five signals, i.e., 3181.57 *m/z*, 3359.10 *m/z*, 5218.25 *m/z*, 6717.05 *m/z*, and 6732.14 *m/z*. The signals of 3181.57 *m/z*, 5218.25 *m/z*, and 6732.14 *m/z* were observed in cluster I spectra but not in cluster II spectra, and those of 3359.10 *m/z* and 6717.05 *m/z* were observed in cluster II spectra but not in cluster I spectra. The absolute intensities of the ions are shown on the *y* axis, and the masses (*m/z*) of the ions are shown on the *x* axis. The *m/z* values represent the mass-to-charge ratio.

As for four *C. rugosa* complex isolates, one *C. pararugosa* isolate was successfully identified by the Bruker Biotyper system but not by Vitek MS (IVD or RUO database). There were six characteristic peaks used to differentiate group I (*C. rugosa*) and group II (*C. pararugosa*): i.e. 3050.6 *m/z*, 3462.3 *m/z*, 5409.0 *m/z*, 6102.2 *m/z* were observed in group I spectra but not in group II spectra, and those of 3131.9 *m/z* and 6363.4 *m/z* (Figures 3A and 3B)

**Figure 3:** Spectra of *C. rugosa* complex isolates. **A.** Two groups of *C. rugosa* complex spectra, i.e., group 1 (*C. rugosa*) and group II (*C. pararugosa*), generated by MALDI-TOF Bruker Biotyper results. **B.** The six characteristic peaks used to differentiate group I (*C. rugosa*) and group II (*C. pararugosa*): i.e. 3050.6 *m/z*, 3462.3 *m/z*, 5409.0 *m/z*, 6102.2 *m/z* were observed in group I spectra but not in group II spectra, and those of 3131.9 *m/z* and 6363.4 *m/z* were observed in group II spectra but not in group I spectra. The absolute intensities of the ions are shown on the *y* axis, and the masses (*m/z*) of the ions are shown on the *x* axis. The *m/z* values represent the mass-to-charge ratio.

## Discussion

Several important findings were demonstrated in this study. First, among the four systems evaluated, only the Bruker Biotyper system could differentiate among three species of *C. parapsilosis* complex and none of the systems could differentiate between the two species of *C. guilliermondii* complex. Second, several characteristic peaks in the spectra by cluster analysis could be used to differentiate between species of the two complex isolates. Third, the performance of identification of *Candida* isolates or of all yeasts isolates by Vitek MS plus SARAMIS system RUO databases was similar to that by Bruker Biotyper system. Finally, the performance of the Phoenix 100 YBC system was better than that of the Vitek 2 Yeast ID system at identifying *Candida* species and all yeasts tested. Both systems had similar results using BAP and SDA media.

The results of the Phoenix Yeast ID system for species-level identification of yeasts (n = 250) and those of the Vitek 2 YST card system were compared with the results of ribosomal ITS sequencing analysis [15]. For all isolates, 94.4% and 89.6% of the isolates were correctly identified by BD Phoenix and Vitek 2, respectively. Considering only the species included in each system's database (n = 245), 96.3% and 91.4% of the isolates were correctly identified by BD Phoenix and Vitek 2, respectively [15]. However, only two isolates of *C. guilliermondii* complex were studied in their study and one was misidentified by Vitek 2 system [15]. In this study, failure of accurate identification of *C. guilliermondii* complex, *R. mucilaginosa* and *C. neoformans* isolates (both BAP and SDA) was the main reason of the poorer performance of Vitek 2 Yeast ID system than that of Phoenix 100 YBC system. *R. mucilaginosa* has also been recognized as an emerging fungal pathogen causing invasive infection [19], [20].

Mancini et al recently compared the performance of the Bruker Biotyper system with that of the Vitek MS system for identification of yeasts [16]. The rate of correct identification to the species level was comparable using the commercial databases (89.8% versus 84.3%; *P* = 0.712). Importantly, the rate of misidentification was significantly higher for Vitek MS (1% versus 12.1%; *P*<0.0001). Our results demonstrated a similar performance by Vitek MS plus SARAMIS system RUO databases as compared with the identification rate reported by Mancin et al [16].

Clinically, separation of three species among *C. parapsilosis* complex isolates is important because of the differences in virulence and antimicrobial susceptibilities [6], [21]. *C. orthopsilosis* had a similar behavior to *C. parapsilosis*, whilst *C. metapsilosis* seems to possess a reduced virulence potential [21]. *L. elongisporus* has been recognized as a yeast species closely related to *C. parapsilosis*. Ahmad et al. showed that currently available phenotypic identification methods (e.g. Vitek 2 system and API 20C) frequently misidentify isolates of *L. elongisporus* as *C. parapsilosis* [22]. However, recent data on small-subunit rRNA gene sequencing have shown that *L. elongisporus* and *C. guilliermondii* should not be included as members of *C. parapsilosis* complex and *C. guilliermondii* complex, respectively [22], [7], [23]. Chen et al demonstrated that *C. guilliermondii* was more commonly isolated from bloodstream infections than *C. fermentati* [40 of 47 (85%) versus 2 of 5 (40%), *P* = 0.043], although *C. fermentati* constituted about 10% of *C. guilliermondii* complex isolates [7], [23]. Moreover, *P. wickerhamii* and *S. salmonicolor* have been reported to cause invasive infection in humans [24], [25].

Westblade et al reported that, based on sequence analysis of the D2 region of the 26S rRNA gene, 97.8% of 852 medically important yeast isolates could be identified to the species level by Vitek MS [26]. Twenty-four isolates (2.8%) were not identified and five isolates (0.6%) were misidentified [26]. Misidentified isolates included one isolate of *C. albicans* identified as *C. dubliniensis*, one isolate of *C. parapsilosis* identified as *C. pelliculosa*, and three isolates of *Geotrichum klebahnii* identified as *Geotrichum candidum*. The rate of correct identification of *C. guillermondii* complex (n = 36) was 97.2% [26]. Our results partly support previous findings [26]–[28].

In the present study, one *C. pararugosa* isolate and three *C. rugosa* isolates were successfully identified by Phoenix 100 YBC (SDA) and Bruker Biotyper. Both the Vitek 2 Yeast ID system (both BAP and SDA) and Vitek 2 MS (IVD and RUO) failed to accurately identify the *C. pararugosa* isolate, even though the Vitek MS (RUO database) contains the spectra of *C. rugosa and C. pararugosa* [8]. *C. rugosa* is a poorly known fungal species in humans [8], [29], [30]. Recently, *C. rugosa* was characterized as a species complex comprising four taxa: *C. rugosa* sensu stricto, *C. pseudorugosa*, *C. neorugosa* and *C. mesorugosa* [8], [29]–[31]. A molecular analysis of the sequences of the D1/D2 domains and the ITS region of the ribosomal genes of 24 clinical isolates phenotypically identified as *C. rugosa* found that 41.6% were identified as *C. pararugosa* [29]. The true prevalence, susceptibility profiles, and clinical roles of these species have not been well elucidated, although *C. rugosa* was reported to be less susceptible to caspofungin compared with other *C. rugosa* complex species [8], [29]–[31].

Several investigators have demonstrated that MALDI-TOF MS could accurately identify all species in *C. neoformans* complex and could differentiate between *C. neoformans* and *C. gattii* [26], [32]. Among the 17 isolates of *C. neoformans* evaluated in our study, all were correctly identified by Bruker Biotyper and Phoenix, and 88.2% by Vitek 2 (SDA). Three isolates of *C. neoformans* complex were not identified by Vitek MS using RUO databases. Although the *C. neoformans* complex isolates tested in this study were not specified to the species level, a previous study showed that only 1% of *C. neoformans* complex isolates were *C. neoformans* var. *gattii (C. gattii*) [33].

In this study, several isolates of commonly encountered yeasts were not correctly identified by either Phoenix 100 YBC or Vitek 2 Yeast ID systems on BAP or SDA, particularly *C. guilliermondii* complex and *C. neoformans* by Vitek 2 Yeast ID system on both BAP and SDA, *C. krusei* by Vitek 2 Yeast ID system on BAP, and *T. asahii* by the Phoenix system on BAP or by the Vitek 2 Yeast ID system on SDA. These misidentifications might have a great impact on clinical management. Two isolates of *C. nivariensis*, a rare but emerging and multidrug-resistant pathogenic yeast [34], were accurately identified by the Bruker Biotyper system. Two C. *zeylanoides* isolates were not correctly identified by either of the systems but one was accurately identified by the Bruker biotyper and Vitek 2 MS (IVD database) systems. This organism has been reported to be associated with bloodstream infections [4].

In this study, using cluster analysis and external validation processes, several characteristic peaks were demonstrated to be useful for differentiating among the three species of *C. parapsilosis* complex. Most importantly, this study is the first to report using characteristic MALDI-TOF MS spectra to separate successfully between *C. guilliermondii* and *C. fermentati*.

In summary, we evaluated the performance of two commercial biochemical identification systems and two MALDI-TOF MS systems for identifying common and rare yeasts. Differences in performance do exist among these systems; however, the differences are not always found in other reports from other laboratories. Regional variations in species distribution of yeasts, various versions of applied database systems, and inconsistent preparation processing of yeasts might contribute to these differences. In clinical microbiology laboratories, MALDI-TOF MS systems present a promising alternative for the identification of not only clinically commonly encountered yeast species, but also several species belonging to *C. parapsilosis* complex, *C. guilliermondii* complex, and *C. rugosa* complex, and other clinically less encountered yeasts.

## References

[1] PfallerM, NeofytosD, DiekemaD, AzieN, Meier-KriescheHU, et al (2012) Epidemiology and outcomes of candidemia in 3648 patients: data from the Prospective Antifungal Therapy (PATH Alliance) registry, 2004–2008. Diagn Microbiol Infect Dis 74: 323–331.2310255610.1016/j.diagmicrobio.2012.10.003

[2] ParmelandL, GazonM, GuerinC, ArgaudL, LehotJJ, et al (2013) *Candida albicans* and non-*Candida albicans* fungemia in an institutional hospital during a decade. Med Mycol 51: 33–37.2268097810.3109/13693786.2012.686673

[3] ChenCY, HuangSY, TsayW, YaoM, TangJL, et al (2012) Clinical characteristics of candidaemia in adults with haematological malignancy, and antimicrobial susceptibilities of the isolates at a medical centre in Taiwan, 2001–2010. Int J Antimicrob Agents 40: 533–538.2300652110.1016/j.ijantimicag.2012.07.022

[4] PereiraGH, MüllerPR, SzeszsMW, LevinAS, MelhemMS (2010) Five-year evaluation of bloodstream yeast infections in a tertiary hospital: the predominance of non-*C. albicans Candida* species. Med Mycol 48: 839–842.2016328110.3109/13693780903580121

[5] HsuehPR, GraybillJR, PlayfordEG, WatcharanananSP, OhMD, et al (2009) Consensus statement on the management of invasive candidiasis in Intensive Care Units in the Asia-Pacific Region. Int J Antimicrob Agents 34: 205–209.1940975910.1016/j.ijantimicag.2009.03.014

[6] BertiniA, De BernardisF, HensgensLA, SandiniS, SenesiS, et al (2013) Comparison of *Candida parapsilosis, Candida orthopsilosis*, and *Candida metapsilosis* adhesive properties and pathogenicity. Int J Med Microbiol 303: 98–103.2340333810.1016/j.ijmm.2012.12.006

[7] ChenCY, HuangSY, TangJL, TsayW, YaoM, et al (2013) Clinical features of patients with infections caused by *Candida guilliermondii* and *Candida fermentati* and antifungal susceptibility of the isolates at a medical centre in Taiwan, 2001–10. J Antimicrob Chemother 68: 2632–2635.2376648610.1093/jac/dkt214

[8] PadovanAC, MeloAS, ColomboAL (2013) Systematic review and new insights into the molecular characterization of the *Candida rugosa* species complex. Fungal Genet Biol 61: 33–41.2416172710.1016/j.fgb.2013.10.007

[9] MarcosJY, PincusDH (2013) Fungal diagnostics: review of commercially available methods. Methods Mol Biol 968: 25–54.2329688310.1007/978-1-62703-257-5_2

[10] LeawSN, ChangHC, SunHF, BartonR, BoucharaJ-P, et al (2006) Identification of medically important yeast species by sequence analysis of the internal transcribed spacer regions. J Clin Microbiol 44: 693–699.1651784110.1128/JCM.44.3.693-699.2006PMC1393093

[11] HsiueHC, HuangYT, KuoYL, LiaoCH, ChangTC, et al (2010) Rapid identification of fungal pathogens in positive blood cultures using oligonucleotide array hybridization. Clin Microbiol Infect 16: 493–500.1962451010.1111/j.1469-0691.2009.02828.x

[12] PutignaniL, Del ChiericoF, OnoriM, MancinelliL, ArgentieriM, et al (2011) MALDI-TOF mass spectrometry proteomic phenotyping of clinically relevant fungi. Mol Biosyst 7: 620–629.2096732310.1039/c0mb00138d

[13] BaderO, WeigM, Taverne-GhadwalL, LugertR, GrossU, et al (2011) Improved clinical laboratory identification of human pathogenic yeasts by matrix-assisted laser desorption ionization time-of-flight mass spectrometry. Clin Microbiol Infect 17: 1359–1365.2094641110.1111/j.1469-0691.2010.03398.x

[14] ChenJH, YamWC, NganAH, FungAM, WooWL, et al (2013) Advantages of using matrix-assisted laser desorption ionization-time of flight mass spectrometry as a rapid diagnostic tool for identification of yeasts and mycobacteria in the clinical microbiological laboratory. J Clin Microbiol 51: 3981–3987.2404853710.1128/JCM.01437-13PMC3838092

[15] PosteraroB, RuggeriA, De CarolisE, TorelliR, VellaA, et al (2013) Comparative evaluation of BD Phoenix and vitek 2 systems for species identification of common and uncommon pathogenic yeasts. J Clin Microbiol 51: 3841–3845.2396650010.1128/JCM.01581-13PMC3889777

[16] ManciniN, De CarolisE, InfurnariL, VellaA, ClementiN, et al (2013) Comparative evaluation of the Bruker Biotyper and Vitek MS matrix-assisted laser desorption ionization-time of flight (MALDI-TOF) mass spectrometry systems for identification of yeasts of medical importance. J Clin Microbiol 51: 2453–2457.2367807110.1128/JCM.00841-13PMC3697679

[17] TengSH, ChenCM, LeeMR, LeeTF, ChienKY, et al (2013) Matrix-assisted laser desorption ionization-time of flight mass spectrometry can accurately differentiate between *Mycobacterium masilliense* (*M. abscessus* subspecies *bolletti*) and *M. abscessus* (sensu stricto). J Clin Microbiol 51: 3113–3116.2382477510.1128/JCM.01239-13PMC3754645

[18] RuanSY, ChienJY, HsuehPR (2009) Invasive trichosporonosis caused by *Trichosporon asahii* and other unusual *Trichosporon* species at a medical center in Taiwan. Clin Infect Dis 49: e11–e17.1948971110.1086/599614

[19] SimonMS, SomersanS, SinghHK, HartmanB, WickesBL, et al (2014) Endocarditis caused by *Rhodotorula* infection. J Clin Microbiol 52: 374–378.2419788810.1128/JCM.01950-13PMC3911467

[20] SpiliopoulouA, AnastassiouED, ChristofidouM (2012) *Rhodotorula* fungemia of an intensive care unit patient and review of published cases. Mycopathologia 174: 301–309.2257694110.1007/s11046-012-9552-9

[21] NémethT, TóthA, SzenzensteinJ, HorváthP, NosanchukJD, et al (2013) Characterization of virulence properties in the *C. parapsilosis* sensu lato species. PLoS One 8 (7): e68704.2387473210.1371/journal.pone.0068704PMC3706360

[22] Ahmad S, Khan ZU, Johny M, Ashour NM, Al-Tourah WH, et al. (2013) Isolation of *Lodderomyces elongisporus* from the catheter tip of a fungemia patient in the Middle East. Case Rep Med 560406. doi: 10.1155/2013/560406. Epub 2013 Apr 3.10.1155/2013/560406PMC363856623653654

[23] CastanheiraM, WoosleyLN, DiekemaDJ, JonesRN, PfallerMA (2013) *Candida guilliermondii* and other species of *Candida* misidentified as *Candida famata*: assessment by vitek 2, DNA sequencing analysis, and matrix-assisted laser desorption ionization-time of flight mass spectrometry in two global antifungal surveillance programs. J Clin Microbiol 51: 117–124.2310035010.1128/JCM.01686-12PMC3536252

[24] NwangumaV, ClevelandK, BaselskiV (2011) Fatal Prototheca wickerhamii bloodstream infection in a cardiac allograft recipient. J Clin Microbiol 49: 4024.2204283110.1128/JCM.05305-11PMC3209132

[25] SharmaV, ShankarJ, KotamarthiV (2006) Endogeneous endophthalmitis caused by *Sporobolomyces salmonicolor* . Eye (Lond) 20: 945–946.1609665910.1038/sj.eye.6702051

[26] WestbladeLF, JennemannR, BrandaJA, BythrowM, FerraroMJ, et al (2013) Multicenter study evaluating the Vitek MS system for identification of medically important yeasts. J Clin Microbiol 51: 2267–2272.2365826710.1128/JCM.00680-13PMC3697678

[27] SendidB, DucoroyP, FrançoisN, LucchiG, SpinaliS, et al (2013) Evaluation of MALDI-TOF mass spectrometry for the identification of medically-important yeasts in the clinical laboratories of Dijon and Lille hospitals. Med Mycol 51: 25–32.2270316410.3109/13693786.2012.693631

[28] Lacroix C, Gicquel A, Sendid B, Meyer J, Accoceberry I, et al. (2013) Evaluation of two matrix-assisted laser desorption ionization-time of flight mass spectrometry (MALDI-TOF MS) systems for the identification of *Candida* species. Clin Microbiol Infect 2013 Mar 7. doi: 10.1111/1469-0691.12210. [Epub ahead of print]10.1111/1469-0691.1221023594150

[29] ParedesK, SuttonDA, CanoJ, FothergillAW, LawhonSD, et al (2012) Molecular identification and antifungal susceptibility testing of clinical isolates of the *Candida rugosa* species complex and proposal of the new species *Candida neorugosa* . J Clin Microbiol 50: 2397–2403.2255323610.1128/JCM.00688-12PMC3405575

[30] ChavesGM, TerçarioliGR, PadovanAC, RosasRC, FerreiraRC, et al (2013) *Candida mesorugosa* sp. nov., a novel yeast species similar to *Candida rugosa*, isolated from a tertiary hospital in Brazil. Med Mycol 51: 231–242.2292892410.3109/13693786.2012.710345

[31] NakagawaY, RobertV, KawarazakiJ, EppingW, SmithMT, et al (2004) Recurrent isolation of an uncommon yeast, *Candida pararugosa*, from a sarcoma patient. Med Mycol 42: 267–271.1528505810.1080/13693780310001597674

[32] PosteraroB, VellaA, CogliatiM, De CarolisE, FlorioAR, et al (2012) Matrix-assisted laser desorption ionization-time of flight mass spectrometry-based method for discrimination between molecular types of *Cryptococcus neoformans* and *Cryptococcus gattii* . J Clin Microbiol 50: 2472–2476.2257359510.1128/JCM.00737-12PMC3405602

[33] LiawSJ, WuHC, HsuehPR (2010) Microbiological characteristics of clinical isolates of *Cryptococcus neoformans* in Taiwan: serotypes, mating types, molecular types, virulence factors, and antifungal susceptibility. Clin Microbiol Infect 16: 696–703.1969476510.1111/j.1469-0691.2009.02930.x

[34] BormanAM, PetchR, LintonCJ, PalmerMD, BridgePD, et al (2008) *Candida nivariensis*, an emerging pathogenic fungus with multidrug resistance to antifungal agents. J Clin Microbiol 46: 933–938.1819978810.1128/JCM.02116-07PMC2268332

